The article "Application of Isothermal Signal Amplification Technique in the Etiological Diagnosis of Gonorrhea and Drug Resistance Gene Detection" was retracted in 2023. Reasons: signs of a paper mill; suspected computer-generated content; unreliable results or conclusions; lack of ethics approval or compliance.

# Application of Isothermal Signal Amplification Technique in the Etiological Diagnosis of Gonorrhea and Drug Resistance Gene Detection

**DOI:** 10.1155/2022/5989889

**Published:** 2022-07-01

**Authors:** Wei Chen, Jinling Zhang, Dongsheng Li, Yue Wang

**Affiliations:** ^1^Wuhan Fourth Hospital, Oncology Department, China; ^2^Wuhan No.1 Hospital, Department of Dermatology, China

## Abstract

*Background:* Isothermal signal amplification technique is developed based on the rolling ring amplification mechanism of cyclic DNA molecules in nature. This technique plays an extremely beneficial role in gonorrhea pathogen identification and drug resistance gene detection. *Aims*: This study analyzes the isothermal signal amplification techniques in the etiological diagnosis of gonorrhea and drug resistance gene detection. *Materials and Methods*: Urethral, cervical secretion, or prostatic fluid samples from 322 cases of gonorrhea collected from January 2018 to December 2021 at the STD clinic of our hospital dermatology department were selected for direct smear examination and gonococcal culture examination; DNA was extracted from urethral, cervical secretion, or prostatic fluid samples and then used for pathogen identification by SAT assay and rolling loop nucleic acid amplification technique, smear examination and pathogen culture examination methods, SAT assay, and isothermal signal amplification technique for comparative sensitivity and specificity analysis. *Results*: The highest rate of gonorrhea positivity was for the urine rolling loop nucleic acid amplification technique, followed by the swab rolling loop nucleic acid amplification technique, and the lowest rate of gonorrhea positivity was for the urine SAT test. The difference in the positivity rate between the two urine testing methods was statistically significant (*P* < 0.05). The highest sensitivity of the urine rolling loop nucleic acid amplification technique method for the detection of gonorrhea pathogens and the lowest sensitivity of the urine SAT method were statistically significant (*P* < 0.01). The differences in sensitivity and specificity between the swab rolling loop nucleic acid amplification technique and the swab SAT method were not statistically significant (*P* > 0.05). ROC curves were plotted based on sensitivity and specificity, with swab SAT assay (*AUC* = 0.998) > rolling loop nucleic acid amplification technique (*AUC* = 0.981). Comparing the negative rates of urine and swab rolling loop nucleic acid amplification technique and urine SAT assay, the differences were not statistically significant (*P* > 0.05). *Conclusion*: The isothermal signal amplification technique improves the shortcomings of gonorrhea pathogen identification means and drug resistance gene detection methods, with good detection sensitivity and specificity, simple operation, low price, and easy promotion, which has obvious advantages in clinical applications and epidemiological studies.

## 1. Introduction

Gonorrhea is difficult to diagnose in patients with nonspecific symptoms, especially in special populations such as women and young children, and may cause complications such as public health problems such as upstream infection of the internal genital system leading to infertility and chronic inflammation that seriously threaten human life and health [1]. Research on the experimental diagnosis, clinical treatment, and epidemiology of this disease has received much attention in recent years [2]. In the diagnosis of gonorrhea, direct smear examination is now commonly used in clinical practice, with the exception of urethral discharge sampling in men with acute urethritis, where the positivity rate can reach 95% [3]. Other lesions and female patients have a low positive rate and have difficulty in identifying different strains with Neisseria [4]. The gonococcal culture test is the gold standard for clinical diagnosis, but it is also influenced by the collection of material and the hypersensitivity of gonococci to antibiotics in the culture medium, and the test cycle is long, time-consuming, and laborious, and the detection rate is very low in asymptomatic and recovering patients [5]. The purity of the sample is required [6]. Therefore, it is still urgent to find and pinpoint the relevant resistance genes, to investigate the mechanisms of drug resistance, and to study the epidemiological characteristics of drug-resistant strains [7].

The isothermal signal amplification technique is a newly developed molecular biology technique based on the amplification mechanism of circular DNA molecules in nature by rolling loops, characterized by the fact that rolling loops can only be replicated in a single-stranded closed state with the presence of corresponding primers in a homothermal rolling [8]. The isothermal signal amplification technique is highly specific and requires low sample purity; if the sample does not contain the target sequence to be detected, the loop probe cannot be looped, and the amplification reaction will not occur [9]. The branched chain amplification effect can increase the sensitivity of detecting mutant molecules to about 10 copies, and its sensitivity is extremely high, and this technique is extremely advantageous in the identification of gonorrhea pathogens and the detection of drug resistance genes [10]. Therefore, the successful implementation of our study will definitely change the current status of gonorrhea diagnosis and treatment, and has excellent market demand and prospects.

## 2. Material and Methods

### 2.1. Research Object

The data of 322 patients admitted to the dermatology and STD clinic of our hospital were analyzed, including 201 males and 121 females, aged 45.6 ± 8.9 years old. Inclusion criteria are as follows: outpatients with suspected urogenital tract infection and informed consent to this study. Exclusion criteria are as follows: cases of prehospital antimicrobial therapy. A total of 322 samples of urinary tract, cervical secretions, or prostatic fluid were collected for direct Smear and Neisseria gonorrhoeae culture, extract DNA from urinary tract, cervical secretion or prostatic fluid, and used SAT test and rolling circle nucleic acid amplification technology to identify pathogenic bacteria. The sensitivity and specificity of the above smear examination and pathogen culture examination methods, SAT detection, and isothermal signal amplification techniques were compared and analyzed to establish an accurate, rapid, and efficient method for the identification of gonorrhea pathogens; to compare and objectively evaluate the advantages and shortcomings of isothermal signal amplification technology in the detection of drug resistance genes in Neisseria gonorrhoeae; and to lay a solid foundation for the optimization of gonorrhea treatment protocols and subsequent research on drug resistance mechanisms. All patients included in this study participated in the study.

### 2.2. Methods

Instruments and reagents are as follows: gonococcal isolation medium was purchased from Zhuhai Yinke Medical Engineering Co. The primers were synthesized by Shanghai Rendu Bioengineering Co., Ltd. and the RNA probe was synthesized by Shanghai Jima Pharmaceutical Technology Co. Ltd.

Specimen collection is as follows: All clinical test specimens were collected from our hospital outpatient clinic. (1) Culture method specimens are as follows: 2-4 cm of secretion from the urethra (urethral swab) of male patients and 0.5-1 cm of mucus from the inner cervical orifice (cervical swab) of female patients were collected with sterile cotton swabs and immediately inoculated with gonococcal selective medium (T-W, incubated at 35 °C in a 5% C02 incubator for 48 h). Round, raised, moist, translucent, or grayish colors were characteristic of gonococci. Oxidase test positive and gram stain negative diplococci were determined as gonococcal positive. (2) In the SAT method specimen, the specimen is not urinated within 2 h before collection, and the first urine sample of about 1 ml is collected and mixed with l ml of urine preservation solution (provided in the kit) to obtain a urine sample, which is frozen at −70 °C for examination.

Sothermal signal amplification technology detection method: sample DNA is extracted, and then a single-stranded oligonucleotide with about 80 bases is designed as a probe, and the probe sequence is fully complementary to the sequence on the gene to be detected. In an environment with low salt ion and ATP levels, T4 ligase binds to the RNA of interest; The pre-designed primers are templated to reproduce the rolling loop to form a single chain of the rolling loop;Another primer amplifies the single-stranded product after binding to the rolling ring, and the amplification sequence is a template for another round of amplified primers; The final product of the reaction is the dsDNA polymorph of various lengths. The amplification flow diagram is shown in Figure 1.

According to the kit instructions, mix 400 *μ*l of the sample with 100 *μ*l of nucleic acid extraction solution, leave it at a constant temperature of 60 °C for 5 min, then leave it at room temperature for another 10 min, and then place it into a semi-automatic nucleic acid extractor for extraction. After the nucleic acid RNA extraction is completed, add 30 l of amplification assay solution (including magnetic beads) to the microreaction tube, prewarm to 42 °C, and generate 100-1000 RNA copies with RNA as the starting template. Each RNA copy is then amplified again and transferred to the photocycliometer 480 fluorescence quantitative PCR instrument to initiate the reaction procedure. PCR instrument to start the reaction program. Reaction procedure is as follows: Carboxyfluorescein was selected for fluorescent labeling, 42 °C for 1 min, 40 cycles; the fluorescent signal was collected once per minute, 40 times in total.

### 2.3. Statistical Analysis

All statistical data of our study were calculated by the statistical processing software as SPSS 25.0. The measurement data were expressed as mean ± standard deviation (X ± SD) using independent samples *t*-test, and the count data were expressed as whole numbers or percentages using Chi-square test. Included data were described by M(QR) if they did not conform to a normal distribution. All statistical tests were two-sided probability tests with a statistical significance of *P* < 0.05.

## 3. Results

### 3.1. Detection of Infection by Different Methods

Urine and swab samples from 322 patients were tested for gonorrhea using SAT and ring-rolling nucleic acid amplification techniques, respectively. The highest rate of gonorrhea positivity was obtained with the urine rolling loop nucleic acid amplification technique, followed by the swab rolling loop nucleic acid amplification technique, and the lowest rate of gonorrhea positivity was obtained with the urine SAT test. The difference in the positivity rate between the two urine assays was statistically significant (*P* < 0.05), while the difference in the positivity rate between the two swab assays was not statistically significant (*P* > 0.05) (see Figure 2).

### 3.2. Evaluation of Testing Methods

The sensitivity of the urine rolling loop nucleic acid amplification technique method was the highest, and the sensitivity of the urine SAT method was the lowest, with a statistically significant difference (*P* < 0.01); the specificity was the opposite, with a statistically significant difference in comparison (*P* < 0.05). The differences in sensitivity and specificity between the swab rolling loop nucleic acid amplification technique method and the swab SAT method were not statistically significant (*P* > 0.05). The differences in sensitivity and specificity between the urine rolling loop nucleic acid amplification technique method and the swab rolling loop nucleic acid amplification technique method were not statistically significant (*P* > 0.05) (see Figure 3).

### 3.3. Sensitivity and Specificity Analysis

ROC curves were plotted according to sensitivity and specificity, and the swab SAT assay (AUC = 0.998) > rolling loop nucleic acid amplification technique (AUC = 0.981), with moderate to high diagnostic accuracy for all of the above assays (see Figure 4).

### 3.4. Assessment of Prognostic Turnaround Rate

There was no significant difference in the negative conversion rates of urine and swab rolling circle nucleic acid amplification technology and urine SAT detection (*P* > 0.05) (see Figure 5).

## 4. Discussion

Early detection of gonorrhea is important for disease control, but the current gonococcal test mainly collects genitourinary secretions as specimens, which can cause painful sampling and reduce the willingness of patients to be tested [11]. In addition, there are shortcomings in sensitivity and specificity. Male patients with gonococcal urethritis usually have more pus in the urethral orifice during the onset of the disease, and positive samples can be detected at the urethral orifice or in the more superficial urethra [12]. In contrast, urethral secretions may be less or absent in those with longer disease duration, which can easily lead to missed detection, and therefore the positive gonococcal detection rate is often low in those with longer disease duration [13].SAT is a noninvasive test that can detect both genitourinary secretions and urine specimens, and collecting urine specimens from the subject for testing not only reduces patient pain but also reduces the workload of clinicians [14]. In the identification of gonorrhea pathogens, secretion smear, pathogenic bacteria culture, and SAT are commonly used in clinical practice [15]. Direct smear examination is limited by sampling and has a low positive rate for lesions other than male acute urethritis secretions and has difficulty in identifying different strains of Neisseria [16]. The SAT method is prone to contamination and false positives and requires high sample purity. As for drug resistance gene detection, although gene sequencing is recognized as an accurate and sensitive detection method, its experimental requirements are high and costly, and the long cycle time is not suitable for clinical studies, especially epidemiological investigations [17]. The isothermal signal amplification technique is a newly developed molecular biology technique based on the amplification mechanism of circular DNA molecules in nature, which is based on the fact that rolling loops can only be replicated in a single-stranded closed state with the presence of corresponding primers in a homothermal rolling [18]. The isothermal signal amplification technique is highly specific and requires low sample purity, while its branched chain amplification effect can increase the sensitivity of detecting mutant molecules to about 10 copies, making it extremely sensitive [19]. This technique is highly advantageous in the identification of gonorrhea pathogens compared to the currently used clinical identification and detection techniques. In terms of drug resistance gene detection, isothermal signal amplification technology is also highly specific and sensitive, but compared to gene sequencing, it is inexpensive, requires low experimental conditions, has a relatively short cycle time, and is easy to promote clinically [20].

The highest rate of gonorrhea positivity in our study was for the urine rolling loop nucleic acid amplification technique, followed by the swab rolling loop nucleic acid amplification technique, and the lowest rate of gonorrhea positivity was for the urine SAT test. The urine rolling loop nucleic acid amplification technique method had the highest sensitivity, and the urine SAT method had the lowest sensitivity for the detection of gonorrhea pathogenic bacteria. Based on sensitivity and specificity, swab SAT assay > rolling loop nucleic acid amplification technique. The culture method has long been the gold standard for detection, but it is not conducive to rapid detection and early diagnosis of gonorrhea pathogens due to the harsh culture conditions, long incubation time, and easy death of isolates [21]. Therefore, nonculture methods are now increasingly used for the diagnosis of gonorrhea pathogens. Among them, isothermal signal amplification is a new nucleic acid detection technique combining the new generation of nucleic acid thermostatic amplification technology and real-time fluorescence detection technology [22]. The basic principle is that a double-stranded DNA copy of the target nucleic acid (RNA) is first generated by M-MLV reverse transcriptase at the same temperature, and then multiple RNA copies are generated from this DNA copy using T7 RNA polymutase [23]. Each RNA copy then enters the next amplification cycle starting from reverse transcription, while a probe with a fluorescent marker specifically binds to these RNA copies to generate fluorescence, which can be captured in real time by a fluorescence detection instrument to reflect the amplification cycle in real time [24]. This method has the advantages of high sensitivity, high specificity, low contamination, and stable reaction. Possible reasons for this are, on the one hand, the low efficiency of SAT assay using the traditional boiling lysis method for nucleic acid extraction, coupled with the high number of inhibitors of SAT assay reactions in the urine composition, resulting in the insensitivity of SAT assay to urine and affecting nucleic acid amplification [25]. In contrast, the isolated culture method, which is the gold standard for the diagnosis of gonorrhea pathogenic bacteria, has high requirements for the environment, collection, and transport of specimens and also may lead to missed detection due to antibiotic use and inactivation of pathogenic microorganisms after inoculation [26]. On the other hand, the isothermal signal amplification technique method uses the magnetic bead method to extract nucleic acid reaction system incorporating a competitive internal standard, thus increasing the sensitivity of the detection reaction [27]. In addition, judging from the ROC curves, the swab isothermal signal amplification technique method and urine isothermal signal amplification technique method have a moderate to high AUC and have a high diagnostic value [28]. And the differences in sensitivity and specificity between urine isothermal signal amplification technique method and swab isothermal signal amplification technique method were not statistically significant, suggesting that both isothermal signal amplification technique method can use urogenital tract secretions and urine as samples to be tested and urine as a noninvasive sampling to avoid the embarrassment and pain of swab sampling in male patients [29]. Therefore, in case of rejection or difficulty in urethral swab sampling in male patients, retention of urine specimens for examination can be considered according to the actual situation, but the concept of first voided urine must be clearly defined at the time of retention of urine specimens, i.e., the time of urine retention must be at least 2 h from the last voided urine, and it must be 30 mL of the first segment of urine [30]. This will ensure accurate and reliable test results. Overall, the isothermal signal amplification technique can exclude false positives caused by dead pathogens at the patient's foci after treatment and the rapid degradation of RNA in dead pathogens, which facilitates the observation of efficacy and judgment of healing after treatment and avoids overtreatment, thus reducing the burden on patients [31].

In conclusion, isothermal signal amplification technology improves the deficiencies of gonorrhea pathogen identification means and drug resistance gene detection methods, has good detection sensitivity and specificity, is simple to operate, is inexpensive and easy to promote, and has obvious advantages in clinical applications and epidemiological studies.

## Figures and Tables

**Figure 1:** Amplification flow model.

**Figure 2:** Different ways to detect infection (in this study, the data of infection detection by different methods were entered into excel software, and the Chi-square test was used for integer representation). The results showed that the difference in the positive rate of the two urine detection methods was statistically significant (*P* < 0.05), while the difference in the positive rate of the two swab detection methods was not statistically significant (*P* > 0.05).

**Figure 3:** Evaluation of testing methods. All the data of evaluation of testing methods in this study were entered into excel software, and the separation and culture method was used as the reference method, and SPSS25.0 was used to calculate the sensitivity, specificity, positive predictive value, and negative prediction of rolling circle nucleic acid amplification technology and SAT method for detecting gonorrhea pathogens value. The results showed that the urine rolling circle nucleic acid amplification method had the highest sensitivity for detecting gonorrhea pathogens, and the urine SAT method had the lowest sensitivity, and the difference was statistically significant (*P* < 0.01); the specificity was opposite, and the difference was statistically significant (*P* < 0.05). There was no significant difference in sensitivity and specificity between the swab rolling circle nucleic acid amplification method and the swab SAT method (*P* > 0.05). There was no significant difference in sensitivity and specificity between urine rolling circle nucleic acid amplification and swab rolling circle nucleic acid amplification (*P* > 0.05).

**Figure 4:** Sensitivity and specificity analysis. All sensitivity and specificity analysis data in this study were entered into excel software, and the separation culture method was used as the reference method. The ROC calculation results using SPSS25.0 showed that the swab SAT assay (AUC = 0.998) > rolling loop nucleic acid amplification technique (AUC = 0.981), with moderate to high diagnostic accuracy for all of the above assays.

**Figure 5:** Assessment of prognostic turnaround rate. All assessment of prognostic turnaround rate data in this study were entered into Excel software, and SPSS25.0 was used for variance calculation. The results showed that there was no statistical difference in the negative conversion rate of urine and swab rolling circle nucleic acid amplification technology and urine SAT detection (significance *P* > 0.05).

## Data Availability

The datasets used and analyzed during the current study are available from the corresponding author upon reasonable request.
